# The “Booster” of Corporate Eco-Innovation: Government Pressure Perceived by Chinese Private Firms

**DOI:** 10.1155/2022/2337867

**Published:** 2022-09-19

**Authors:** Changbo Li

**Affiliations:** School of Management and Engineering, Nanjing University of Information Science & Technology, Nanjing 210044, China

## Abstract

This study explores the relationship between perceived government pressure for environmental regulation and corporate eco-innovation. Based on the questionnaire data of Chinese private firms in 2016, this study explores the role of government pressure perceived by private firms in corporate environmental innovation, and the moderating effects of foreign ownership and entrepreneurs' political status. The results show that there is a positive relationship between perceived government environmental regulatory pressure and corporate eco-innovation, and this relationship can be strengthened by foreign ownership and entrepreneurs' political status. These findings provide a new strategic motivation for firms to undertake eco-innovation, i.e., the environmental regulatory pressure released by the government can urge firms to undertake strategies as an external “booster.”

## 1. Introduction

In recent years, environmental issues have received increasing attention from the Chinese government and various business stakeholders. From the government's proposal that “green water and green mountains are the silver mountain of gold” and its strong advocacy of corporate environmental protection and pollution reduction, to the implementation of the “Plastic Restriction Order” and further interpretation of corporate eco-innovation, all reflect China's new requirements for corporate environmental responsibility. Different scholars have given different explanations for the so-called eco-innovation. OECD considers environmental innovation as “any innovative activity that reduces environmental impact” [1], while Europeia considers environmental innovation as a progress of sustainable development [2]. According to Kemp and Pearson [3], eco-innovation refers to the production, development, or absorption of relevant alternatives that can reduce environmental risks, pollution, or other negative impacts [4]. In order to meet the growing economic demands and address the growing environmental problems, China has developed many environmental policies [5]. In this new era, the government requires firms to not only reduce pollution, but also to reduce pollution from another perspective – by proactively reducing emissions through eco-innovation, thereby achieving sustainable development.

Many scholars have studied the motivation of corporate eco-innovation, some of which consider corporate eco-innovation as a strategic behavior of firms [6], while others suggest that government intervention affects the process of eco-innovation [7–9]. In addition, technology is one of the important factors that promote environmental innovation in firms [10, 11]. Firms' own technological capabilities, external market influences, and consumer demands all influence corporate green innovation. However, relatively few studies have examined firms' innovative behavior through entrepreneurs' perceptions of government pressure on environmental regulatory [5]. In order to fill the existing research gap, we should clarify why entrepreneurs engage in corporate eco-innovation when they perceive pressure from government. Institutional theory can be a good solution to this problem. It suggests that entrepreneurs and firms tend to do what the government expects if they want to achieve sustainable development. In China's institutional context, the key resources available to firms are controlled by the government and firms must meet the government's expectations.

Based on these literature reviews and the research gaps described above, the purpose of this study is clear: What impact do entrepreneurs have on the eco-innovation of firms when they feel the pressure of government regulation? Furthermore, what role does the self-perceived political status of the entrepreneur and the foreign ownership of the firm play in this influence process? Based on these research gaps, we used cross-sectional data from 2,244 Chinese private firms in 2015 to address this question by examining the environmental regulatory pressures felt by entrepreneurs and how this affects firms to innovate environmentally. According to previous literature, firms heed the government's calls or “orders” to maintain their political legitimacy in Chinese institutional context. In addition, we argue that entrepreneurs' perceived pressure is positively related to firms' environmental behavior. Furthermore, by considering the moderating role of entrepreneurs' political connections and foreign ownership in the firm, this study provides a more accurate framework for the relationship between the role of government and corporate eco-innovation in the unique Chinese institutional context. Thus, this study provides new evidence on why some firms are willing to engage in eco-innovation and why the political status of entrepreneurs and foreign ownership of firms significantly influence corporate environmental strategies.

In order to answer the above research questions, this study provides several contributions to the current literature on corporate eco-innovation. First, this study uses institutional theory to examine the response of firm behavior to perceived governmental environmental regulatory pressures, combining “perceived pressures” with “corporate eco-innovation”. Second, it gives explanations for the factors affecting firm eco-innovation, both internal and external, using the entrepreneurs' own political connections and the firm's foreign ownership as moderating variables. This also brings valuable practical insights and implications for researchers and policy makers.

The remainder of this study is organized as follows.  Section 2 provides further details on the theoretical framework of the study and sets out three hypotheses of this study. The third section describes the data and the methodology of analysis. The empirical results are then presented, and next section shows our discussions and limitations. Conclusions are outlined in the final section.

## 2. Theories and Hypotheses

### 2.1. Relationship between Government Pressure and Eco-Innovation

Eco-innovation has become an important part of green economy. Among the existing studies, there is no shortage of research on corporate eco-innovation. Most scholars focus on a resource-based perspective with institutional and stakeholder theories as the underlying logic, and their drivers are mostly external non-institutional factors, such as markets and monitoring [4]. Institution is defined as “regulatory, normative, and cognitive structures and activities that provide stability and meaning to social behavior” [12]. In the Chinese context, the policies proposed by the government are considered to be an institutional regulation. Institutional theory suggests that institutionalized activities have an impact on individuals, organizations, and interorganizations [13]. At the individual level, managers consciously or unconsciously follow norms, habits, customs, and traditions [14]. At the organizational level, shared political, social, cultural, and belief systems support traditions of institutionalized activities. At the interorganizational level, pressure from government determines what is socially acceptable and expected organizational behavior [15]. That is, firms make decisions under external pressure. Therefore, we can assume that when firms feel environmental regulatory pressure from the government, they tend to follow the government's instructions. Therefore, we propose the following hypothesis:

**Hypothesis 1 .**

The greater the perceived government pressure on environmental regulation, the more firms will engage in corporate eco-innovation.

### 2.2. Moderation Effect of Political Status

In the process of business operation, many firms have some political linkages with the government, which can influence corporate strategies to some extent, such as charitable donations, green economy. When an entrepreneur perceives that he has a high political status (by comparing with people around him or others), he may participate in some government organizations, such as being a deputy to the National People's Congress or a member of the Chinese People's Political Consultative Conference. These positions influence their business behavior. In other words, they are more willing to be close to the government and more inclined to follow the government's wishes. Therefore, the higher the political status of entrepreneurs, the closer the relationship between firms and the government. Under the such logic, the closer the entrepreneur's relationship with the government, the more willing the firm is to follow the government's instructions or meet its expectations, so it is more willing to engage in eco-innovation. Therefore, we propose the following hypothesis:

In China, the government controls key resources needed by firms to develop. As the provider of resources, local governments provide relevant resources to local firm through government intervention [16–18]. As mentioned above, under institutional pressure, individuals tend to follow norms, while firms under pressure will follow government directives in order to gain “legitimacy” [19, 20]. Thus, when the entrepreneur has a certain status in society, he has more personal contact with the government. When the entrepreneur perceives more pressure, he is more willing to follow the new requirements for environmental protection and to do eco-innovation. For example, firms are more willing to make charitable donations when entrepreneurs have more connections to the government [21]. Therefore, based on this logic, firms with higher political status of entrepreneurs are more likely to be perceived by local governments to engage in eco-innovation. At the same time, this behavior will help firms obtain resources from local governments more easily through corporate environmental strategies. Therefore, we propose Hypothesis 2:

**Hypothesis 2 .**

The entrepreneur's perceived political status strengthens the positive relationship between government pressure and corporate eco-innovation.

### 2.3. Moderation Effect of Foreign Ownership

A high proportion of foreign ownership is becoming more and more common in the operation of modern firms. The higher proportion of foreign ownership means that firms are more international. They are more willing to align themselves with international standards in terms of business practices or top management than to follow government arrangements, which means that they are increasingly operating outside the government. Thus, these firms lack a certain degree of “legitimacy” in their domestic operations. At this point, such firms need to follow the instructions and ideas of the government. For example, when they feel the pressure of government environmental regulation, they should engage in eco-innovation to gain government legitimacy.

When the foreign ownership is high, we can assume that the firm is more international, which means that the firm lacks a certain local background or political connection to the local government during its operations. In the Chinese context, where the government controls the main resources needed for business activities, foreign firms have relatively little legitimacy in their operations due to their lack of association with the government compared with local firms. Entrepreneurs will face more serious pressure from government environmental regulation, and they need to make more pro-government behavior in order to gain resources from the government [22]. Thus, when firms have a higher foreign ownership, they will be more willing to do eco-innovation for the sake of legitimacy in order to gain the government's perception and attention, and thus easier access to government resources. Therefore, we propose Hypothesis 3:

**Hypothesis 3 .**

Foreign ownership strengthens the positive relationship between government pressure and corporate eco-innovation.

## 3. Methodology

### 3.1. Data and Sample

In order to study the impact of perceived government pressure for environmental regulation on corporate eco-innovation, we used a questionnaire data describing Chinese private firms. The questionnaire comes from the private firm research group consisting of the Chinese Central United Front Work Department, the All-China Federation of Industry and Commerce, the State Administration for Industry and Commerce, and the China Private Economy Research Association. The research group conducts a nationwide sample survey on the status of private firms every two years, and its time span has exceeded over 20 years. From the previous surveys, the data obtained each time can accurately reflect the basic situation of China's private economy and the difficulties and problems encountered in its development. This study uses data from the 12th survey conducted by the research group in 2016, and this source of data has been confirmed in many previous literature [23–25].

The survey respondents are all private entrepreneurs in China. The survey collected data covering more than 8,000 firms. However, due to the lack of some survey data and the limitation of questionnaire completeness, some data were not included in the analysis. We ended up with a final sample of 2,244 observations.

### 3.2. Variable Measurements

Corporate eco-innovation, our dependent variable in this study, is measured by the probability of innovation, which is a dummy variable, and firms with eco-innovation in 2015 are coded as 1, and otherwise 0 [26].

Government pressure perceived by firms for environmental regulation, the independent variable of this study, is measured by the Likert 5-point scale. The variable values 1 for firms with no perceived government pressure and values 5 for firms with highest degree of perceived government pressure.

Political status presents the entrepreneur's self-perceived status ladder compared with their peers in society. The variable is measured by 10 scales, 1 being the lowest and 10 being the highest. Political status is widely used in corporate strategies literature and is considered an important driver influencing their nonmarket strategies [27].

The variable foreign ownership refers to the proportion of foreign capital including Hong Kong, Macao and Taiwan parts in the net assets of firms in the current operation process. The higher the proportion, the more foreign capital is invested in the firms' operation, while domestic capital is relatively less. Firms with high degree of foreign ownership are more closely connected with foreign investors and has relatively less tied to the stakeholders in China, and firms will encounter more serious legitimacy challenges in operating in China [28].

In this study, we follow the previous literature and control for a number of variables at two levels. First, at the entrepreneurial level, the entrepreneur's gender, age, education level, salary, and political connection are all considered as important influences on corporate strategies. Studies have shown that firms with more female executives are more willing to innovate when faced with environmental problems [29]. Older executives are more conservative when confronted with innovation [30]. The variable gender is measured as 1 for males and 0 for females. The variable age is calculated as the difference between the entrepreneur's year of birth and 2016. The variable salary is calculated as the natural logarithm value of the actual entrepreneurial annual salary. The entrepreneurial education and foreign education experience are controlled in the analysis. The variable education is measured as 1 for junior high school and below, 2 for senior high school, 3 for junior college, 4 for undergraduate degree, 5 for master degree, and 6 for doctorate degree. Foreign education is a dummy variable, coded as 1 for overseas education experience, and 0 otherwise. Political connection is well considered by most previous studies as a key factor that affects corporate nonmarket strategies [31]. In this study, political connection is a dummy variable coded as 1 if the entrepreneur is a deputy of the National People's Congress or a member of the Chinese people's Political Consultative Conference, and 0 otherwise. In addition, we included the variable charity member, measured as 1 for entrepreneurs participating in charity organizations, and 0 otherwise.

At the firm level, firm size is considered to be one of the most important factors influencing a firm's environmental behavior, since larger firms are more flexible in resource usage in environmental innovation [32]. In this study, firm size is measured as the natural logarithm value of a firm's total employees. Firm age is measured as the number of years a firm has been in existence until the end of 2016. The studies have proved that firms with a longer history have a higher social relevance and they are more active in the face of environmental innovation [33]. Also, corporate performance affects their environmental behavior, and previous studies have proved that firms with good performance are more likely to practice corporate environmental practices [34]. We measure the performance as the value of Return to Assets (ROA). Finally, we include industrial dummies and regional dummies to control for the potential industrial and regional variances.

## 4. Results

### 4.1. Descriptive Statistics and Correlations

Table 1 reports sample characteristics, including sample size, mean, and standard deviation of each variable. It can be seen that the sample includes 2,244 private firms, of which 17% have made eco-innovation, and the mean value and standard deviation of each variable are within the acceptable range.

Table 2 summarizes the Pearson correlation analysis results of all variables in this study. It can be seen that the government pressure is positively correlated with eco-innovation (0.18), which is in line with expectations, and the first inertia between any two variables is not higher than 0.5. Therefore, there is little concern about the high correlations between variables. At the same time, the variance inflation factor (VIF) is calculated and can be found that the highest VIF value is 1.95, and the average VIF value is 1.25, which are lower than the critical value of 10 as a general requirement [35]. Therefore, the collinearity interference will not be a significant problem in this analysis.

### 4.2. Hypotheses Tests

Table 3 reports the probit model regression results of this analysis. Model (1) only adds all control variables. Model (2) adds the independent variable. Model (3) adds the first moderating variable and its interaction item (Political status × Government pressure), and Model (4) adds the second moderating variable and its interaction item (Foreign ownership × Government pressure). Model (5) adds all variables to test the three hypotheses together.

Hypothesis 1 proposes that entrepreneurs' perceived government pressure on environmental regulation promotes corporate eco-innovation. In Model (2), it can be seen that the coefficient of government pressure is 0.154 with *p* value of less than 0.01, which is positive and significant. Therefore, we can verify the positive impact of government pressure on corporate eco-innovation. Therefore, Hypothesis 1 is supported.

Hypothesis 2 proposes that entrepreneurs' self-perception of political status plays a positive moderating role in the main hypothesis. In Model (3), it can be seen that the coefficient of the interaction term between political status and government pressure is 0.026, with *p* value of less than 0.05, which is positive and significant. It means that the higher the political status of entrepreneurs' self-perception, the positive impact of government pressure on corporate eco-innovation will be enhanced. Therefore, Hypothesis 2 is supported.

Hypothesis 3 proposes the positive moderating effect of foreign ownership. In Model (4), the coefficient of the interaction term between foreign ownership and government pressure is 0.01 with *p* value of less than 0.05, which is positive and significant. It can be seen that the higher the proportion of foreign ownership, the stronger the positive impact of government pressure on corporate eco-innovation. Therefore, Hypothesis 3 is also supported.

## 5. Discussions

The purpose of this study is to explore the relationship between government pressure on environmental regulation perceived by entrepreneurs and corporate eco-innovation, as well as the moderating effects of political status and foreign ownership. By empirically testing the data from the 12th national private firms survey in 2016, we find that government pressure has a significant impact on corporate eco-innovation. Specifically, the more perceived pressure of environmental regulation from the government, the more firms are able to promote eco-innovation. This result supports our hypothesis about firms' motivates to undertake eco-innovation. Meanwhile, based on the institutional theory, entrepreneurs will be willing to “listen to the government” when they perceive certain government pressure in order to gain legitimacy for sustainable operations and better performance. Thus, firms with high degree of political status and more foreign ownership have more incentives to engage in eco-innovation to obtain necessary resources and legitimacy controlled by the government.

### 5.1. Contributions and Implications

This study contributes to the existing literature in several aspects. First, to the best of our knowledge, this study is one of the few empirical studies to examine the relationship between government pressure on environmental regulation perceived by firms and corporate eco-innovation. More precisely, this study is the first to focus on its direct relationship. Considering that the particular factor of institution plays an important role in this relationship, institution theory is proposed in the context of eco-innovation research. Thus, this study broadens the scope of corporate eco-innovation and entrepreneurs' perception of government pressure.

Second, based on previous literature, we find that entrepreneurs' political status plays an important role in corporate environmental practices, and positively moderates the positive relationship between government pressure and corporate eco-innovation. Institutional theory has previously noted the role of the government in shaping corporate nonmarket strategies [36, 37]. In this study, we have expanded the political status of entrepreneurs. Instead of using the previous dummy variables such as deputies to the National People's Congress and members of the Chinese People's Political Consultative Conference, we explore the dual political pressure regulation of self-perceived political status on external pressure from the perspective of entrepreneurs. Therefore, using the Chinese context, our study finds that China can better reveal the influence of institutional environment on corporate environmental behavior.

### 5.2. Limitations and Future Research Directions

There are some limitations to our study, which provides a direction for future research. First, although we have clearly explained the motives of firms to engage in eco-innovation from the perspective of institutional theory, these motives still depend on political relevance. Some scholars pointed out that there are other motives for corporate eco-innovation, rather than purely political considerations [38, 39]. Future research needs to further test whether political concerns are indeed the main motivation for firms to engage in eco-innovation.

Second, our study measures corporate environmental behavior in terms of whether they engage in eco-innovation, which captures firms' willingness but not the intensity of their eco-innovation. Thus, it cannot well explain the changes in the intensity of corporate eco-innovation. Future research may find a better way to measure the intensity of corporate eco-innovation and thus better explore the dynamics of this variable.

Third, from the perspective of institutional pressure, we test the positive relationship between government pressure and corporate eco-innovation, and assume that firms can gain legitimacy from the government through eco-innovation. Previous studies have demonstrated that firms engaged in corporate eco-innovation are more likely to gain access to government resources, but the performance benefits brought by government legitimacy are not clear. Research on these issues may provide greater insight into the impact of corporate eco-innovation on firm benefits. Therefore, how to gain government legitimacy through corporate environmental innovation, which leads to better benefits, is an important topic for future research.

## 6. Conclusions

The analysis of the data on the 12th Chinese private firms survey conducted by the private enterprise research group composed of the Central United Front Work Department, the All-China Federation of Industry and Commerce, the State Administration for Industry and Commerce, and the China Private Economy Research Association provides better evidence of the influence of institutional environment on firm behavior, especially when entrepreneurs feel more pressure from the government in terms of environmental regulation, firms will be more willing to engage in eco-innovation. Political status and foreign ownership are important factors. As a complement to “legitimacy”, both play the positive moderating effects. We hope that this study will contribute to a better understanding of the factors influencing corporate eco-innovation, especially from the perspectives of institutional aspects.

## Figures and Tables

**Table 1:** Characteristics of the sample.

	N	Mean	S. D.	*P*1	P99
Eco-innovation	2,244	0.17	0.38	0	1
Government pressure	2,244	2.51	1.28	1	5
Gender	2,244	0.82	0.38	0	1
Age	2,244	45.89	9.47	25	67
Education	2,244	2.98	1.13	1	6
Foreign education	2,244	0.13	0.34	0	1
Salary	2,244	3.18	1.43	0	7.67
Political connection	2,244	0.33	0.47	0	1
Charity member	2,244	0.2	0.40	0	1
Firm size	2,244	3.56	1.81	0	7.78
Firm age	2,244	10.5	6.66	1	30
ROA	2,244	7.64	233.76	−1	3.62

**Table 2:** Correlation matrix of variables.

Variables	(1)	(2)	(3)	(4)	(5)	(6)	(7)	(8)	(9)	(10)	(11)	(12)
(1) Eco-innovation	1.00											
(2) Government pressure	0.18	1.00										
(3) Gender	0.07	0.05	1.00									
(4) Age	0.11	0.07	0.12	1.00								
(5) Education	0.16	−0.01	0.04	−0.15	1.00							
(6) Foreign education	0.07	0.01	0.01	−0.04	0.22	1.00						
(7) Salary	0.15	0.08	0.11	0.09	0.17	0.10	1.00					
(8) Political connection	0.19	0.09	0.11	0.29	0.20	0.10	0.23	1.00				
(9) Charity member	0.13	0.02	0.07	0.04	0.14	0.08	0.18	0.17	1.00			
(10) Firm size	0.31	0.16	0.18	0.26	0.35	0.13	0.39	0.49	0.24	1.00		
(11) Firm age	0.16	0.11	0.09	0.40	0.12	0.07	0.22	0.36	0.13	0.48	1.00	
(12) ROA	−0.01	0.01	−0.02	−0.04	−0.02	−0.01	−0.01	−0.02	−0.01	−0.02	−0.03	1.00

**Table 3:** Regression results.

	(1)	(2)	(3)	(4)	(5)
	Eco-innovation	Eco-innovation	Eco-innovation	Eco-innovation	Eco-innovation
Gender	−0.004	−0.015	−0.026	0.035	0.029
	(0.103)	(0.103)	(0.104)	(0.123)	(0.124)
Age	0.005	0.006	0.005	0.004	0.003
	(0.004)	(0.004)	(0.004)	(0.005)	(0.005)
Education	0.121^*∗∗∗*^	0.131^*∗∗∗*^	0.127^*∗∗∗*^	0.139^*∗∗∗*^	0.140^*∗∗∗*^
	(0.035)	(0.036)	(0.036)	(0.042)	(0.042)
Foreign education	0.113	0.130	0.101	0.135	0.090
	(0.098)	(0.098)	(0.100)	(0.116)	(0.118)
Salary	0.059^*∗∗*^	0.052^*∗∗*^	0.045^*∗*^	0.063^*∗∗*^	0.054^*∗*^
	(0.025)	(0.026)	(0.026)	(0.029)	(0.030)
Political connection	0.102	0.092	0.045	−0.019	−0.090
	(0.081)	(0.081)	(0.084)	(0.096)	(0.1)
Charity member	0.246^*∗∗∗*^	0.262^*∗∗∗*^	0.278^*∗∗∗*^	0.320^*∗∗∗*^	0.325^*∗∗∗*^
	(0.082)	(0.083)	(0.084)	(0.097)	(0.098)
Firm size	0.147^*∗∗∗*^	0.137^*∗∗∗*^	0.137^*∗∗∗*^	0.168^*∗∗∗*^	0.166^*∗∗∗*^
	(0.027)	(0.028)	(0.028)	(0.033)	(0.033)
Firm age	−0.001	−0.002	−0.004	0.003	0.001
	(0.006)	(0.006)	(0.006)	(0.007)	(0.008)
ROA	0.000	0.000	0.000	0.000	0.000
	(0.001)	(0.001)	(0.001)	(0.001)	(0.001)
Government pressure		0.154^*∗∗∗*^	0.015	0.151^*∗∗∗*^	0.020
		(0.028)	(0.071)	(0.034)	(0.083)
Political status			−0.030		−0.013
			(0.039)		(0.047)
Political status × Government pressure					
			0.026^*∗∗*^		0.024
			(0.013)		(0.015)
Foreign ownership				−0.040^*∗∗*^	−0.029
				(0.020)	(0.020)
Foreign ownership × Government pressure					
				0.010^*∗∗*^	0.007
				(0.005)	(0.005)
Industrial dummies	Included	Included	Included	Included	Included
Regional dummies	Included	Included	Included	Included	Included
Constant	−2.489^*∗∗∗*^	−2.943^*∗∗∗*^	−2.725^*∗∗∗*^	−3.115^*∗∗∗*^	−3.043^*∗∗∗*^
	(0.377)	(0.392)	(0.435)	(0.458)	(0.514)
Observations	2,244	2,244	2,192	1,738	1,705
Pseudo *R*^2^	0.178	0.193	0.199	0.228	0.235

*Note.* Standard errors are in parentheses, ^*∗∗∗*^*p* < 0.01, ^*∗∗*^*p* < 0.05, ^*∗*^*p* < 0.1.

## Data Availability

The second-hand survey data used to support the findings of this study were supplied by the Chinese Academy of Social Sciences under license and so cannot be made freely available. Requests for access to these data should be made to the author Peng Lv, lv-peng@cass.org.cn.
